RETRACTED

# Chemotherapeutic Potential of 2-[Piperidinoethoxyphenyl]-3-Phenyl-2H-Benzo(b)pyran in Estrogen Receptor- Negative Breast Cancer Cells: Action via Prevention of EGFR Activation and Combined Inhibition of PI-3-K/Akt/FOXO and MEK/Erk/AP-1 Pathways

**DOI:** 10.1371/journal.pone.0066246

**Published:** 2013-06-19

**Authors:** Ruchi Saxena, Vishal Chandra, Murli Manohar, Kanchan Hajela, Utsab Debnath, Yenamandra S. Prabhakar, Karan Singh Saini, Rituraj Konwar, Sandeep Kumar, Kaling Megu, Bal Gangadhar Roy, Anila Dwivedi

**Affiliations:** 1 Division of Endocrinology, CSIR-Central Drug Research Institute, Lucknow, Uttar Pradesh, India; 2 Medicinal and Process Chemistry, CSIR-Central Drug Research Institute, Lucknow, Uttar Pradesh, India; 3 Department of Surgery, King George’s Medical University, Lucknow, Uttar Pradesh, India; 4 Institute of Nuclear Medicine and Allied Sciences, DRDO, Delhi, India; Florida International University, United States of America

## Abstract

Inhibition of epidermal growth factor receptor (EGFR) signaling is considered to be a promising treatment strategy for estrogen receptor (ER)-negative breast tumors. We have investigated here the anti-breast cancer properties of a novel anti-proliferative benzopyran compound namely, 2-[piperidinoethoxyphenyl]-3-phenyl-2H-benzo(b)pyran (CDRI-85/287) in ER- negative and EGFR- overexpressing breast cancer cells. The benzopyran compound selectively inhibited the EGF-induced growth of MDA-MB 231 cells and ER-negative primary breast cancer cell culture. The compound significantly reduced tumor growth in xenograft of MDA-MB 231 cells in nude mice. The compound displayed better binding affinity for EGFR than inhibitor AG1478 as demonstrated by molecular docking studies. CDRI-85/287 significantly inhibited the activation of EGFR and downstream effectors MEK/Erk and PI-3-K/Akt. Subsequent inhibition of AP-1 promoter activity resulted in decreased transcription activation and expression of c-fos and c-jun. Dephosphorylation of downstream effectors FOXO-3a and NF-κB led to increased expression of p27 and decreased expression of cyclin D1 which was responsible for decreased phosphorylation of Rb and prevented the transcription of E2F- dependent genes involved in cell cycle progression from G1/S phase. The compound induced apoptosis via mitochondrial pathway and it also inhibited EGF-induced invasion of MDA-MB 231 cells as evidenced by decreased activity of MMP-9 and expression of CTGF. These results indicate that benzopyran compound CDRI-85/287 could constitute a powerful new chemotherapeutic agent against ER-negative and EGFR over-expressing breast tumors.

## Introduction

Breast cancer is the most common cancer diagnosed in women and the second most common cause of female cancer- related deaths [1]. The anti-hormones are suitably used for therapy of ER- positive breast cancer patients [2], [3]. In contrast to ER- positive, the ER- negative (ER-) breast cancers that constitute about 30% of the total, lack the E2-ER-ERE mediated hormone-dependent cell-proliferation pathway [4]. In ER- negative tumors, overexpression of EGFR or HER-2, leading to increased growth factor signaling, is observed [5]. A subgroup of ER-negative tumors is also negative for the expression of progesterone receptor and HER-2 protein [6]. Such tumors are designated as ‘triple-negative’ and are characterized by their unique molecular profile, aggressive behavior and distinct patterns of metastasis. Overexpression of the epidermal growth factor family of receptors (EGFR) in ER- ve cells has been the basis for the implication of EGF-induced mitogenic signal for the enhanced proliferation of these cancer cells [7], [8]. Hence, EGFR could serve as a target for therapeutic intervention in a subgroup of triple-negative breast cancer patients.

RETRACTED

Major pathways associated with EGFR signaling include the Ras/MAPK pathway, the phosphatidyl inositol 3-kinase (PI3K)/Akt pathway, the Janus kinase (JAK)/signal transducers and activators of transcription. These signaling pathways ultimately affect cell proliferation, survival, motility, and adhesion [1]. Thè key survival pathway modulated by EGFR is the MEK/Erk kinase cascade [9] which exerts its mitogenic and invasive effects via AP-1 transcriptional complex [10]. AP-1 transcription factors are believed to be responsible for cellular proliferation as well as invasion of ER-negative breast cancer cells [11]. EGF also exerts mitogenic effects by activating NF-κB and deactivating Forkhead transcripton factor FOXO-3a via activation of PI-3-K/Akt - dependent signal transduction pathway. The activated NF-κB up-regulates the expression of the cell cycle regulatory ccD1 gene that induces phosphorylation of Rb and cell-cycle progression and it also upregulates anti-apoptotic genes BclxL and XIAP [12]. Studies in mammalian cells have shown that the activation of FOXO-3a induces cell cycle arrest and/or apoptosis through the up-regulation of its key target genes such as p27^Kip1^, Bim, Bclxl and XIAP [13]. EGF has been shown to stimulate the migration of both normal and tumor cells [14]. It has been established that both Akt and Erk cell survival pathways mediate EGF- induced invasion of breast cancer cells via induction of MMP-9 activity [15].

At CDRI, based on structure-activity relationship, 2-[piperidinoethoxyphenyl]-3-phenyl-2H-benzo (b) pyran (CDRI-85/287) was synthesized as possible anti-cancer and antiestrogenic agent [16], [17]. The compound displays significant anti-estrogenic activity and inhibits uterine growth, as is evident from earlier studies carried out in ovariectomized rats [18], [19] and also interferes with the formation of estrogen- ER complex [20]. The compound has also shown anti-estrogenic potential at uterine level in rhesus monkeys [21]. Further, CDRI-85/287 has shown significant anti-proliferative activity in endometrial cancer cells via inhibition of estrogen receptor pathway and cell survival pathway [22]. Cytotoxic effects of benzopyran based platinum II complexes have been reported earlier in ER- negative breast cancer cells but their mechanism of action have not been explored in these cells [23].We hypothesized that compound may interfere with various signaling mechanisms and inhibit growth in breast cancer cells which do not express ER. In this context, we report here the anti-proliferative activity of benzopyran derivative CDRI-85/287 in ER- negative breast cancer cells. The study demonstrates that CDRI-85/287 exerts its anti-proliferative and anti-invasive properties in ER negative breast cancer cells via preventing EGFR activation and subsequently inhibiting the tumor growth via inhibition PI-3-K/Akt and MEK/Erk pathways. The potent in vitro and in vivo anti-tumor activity of this compound in ER- negative breast cancer cells showed that CDRI-85/287 can serve as a lead candidate molecule for development of efficacious anti-breast cancer agent for the management of disease in patients with EGFR - overexpressing breast tumors.

RETRACTED

## Materials and Methods

### Compound

2-[piperidinoethoxyphenyl]-3-phenyl-2H-benzo(b) pyran (CDRI-85/287), was synthesized according to the methods as described earlier [18]. Fig. 1A shows the chemical structure of the compound.

**Figure 1:** Anti-proliferative activity of CDRI-85/287 in ER-negative breast cancer cells. (A) Structure and molecular formula of CDRI-85/287. (B) CDRI-85/287 suppresses the growth of ER-negative and EGFR over-expressing breast cancer cells MDA-MB231 and primary breast adenocarcinoma cells. Cells were treated with indicated concentrations of compound for 48h in the absence or presence of 100 ng/ml of EGF. Cell viability was measured using MTT cell viability assay. The percentage of viable cells was calculated as the ratio of treated cells to the control cells. Results are expressed as mean ± SEM, n = 5. p values are a-p<0.001, b<0.01, c-p<0.05 and d-p>0.05 vs. control and e-p<0.001, f-p<0.01, g-p<0.05, h-p>0.05 vs. EGF.

### Cell lines and cell culture

Human breast cancer cell line, MDA-MB 231 and normal kidney cell lines HEK-293 and VERO were purchased from American Type Culture Collection (Manassas, VA, USA). Cells were maintained in DMEM supplemented with 10% fetal bovine serum (FBS). Cells were cultured at 37°C and 5% CO_2_. Prior to experiments, cells were cultured in phenol red-free DMEM supplemented with 10% charcoal stripped fetal bovine serum.

RETRACTED

### Primary cell culture of breast adenocarcinoma

Breast carcinoma samples were collected in the operating room of the Department of Surgery, King George’s Medical University, Lucknow. A specific written informed consent was obtained from patients, and the study was approved by the Institutional Ethics Committee, King George’s Medical University, Lucknow, India. The breast cancer tissue was collected from 60-65 year old post-menopausal women suffering from infiltrating ductal carcinoma in breast with high grade lesion and metastasis. Pathological report showed that the samples were negative for ER and PR expression and positive for EGFR.

The cell isolation was based on the methods of Bresch et al., 1983 [24]. Briefly, tissue were collected in DMEM, minced in 1-mm pieces, and incubated with 1 mg/ml collagenase and DNase (2 mg/ml) in DMEM for 2 h at 37°C with periodic mixing. Digested tissue was mechanically dissociated through a 1-ml tip and resuspended in 10 ml of fresh DMEM. The cells were separated from tissue clumps and debris by decantation and centrifugation, washed twice with DMEM containing 10% fetal bovine serum, 1 mM sodium pyruvate, 2 mM L-glutamine, and 2% of antibiotic-antimycotic solution (Sigma-Aldrich, USA) and then transferred into plastic culture flasks (75 cm2, Corning, USA). Cells were incubated at 37 °C with saturating humidity and 5% CO2. Prior to experiments, cells were cultured in phenol red-free DMEM supplemented with 10% charcoal stripped fetal bovine serum and 1% antibiotic antimycotic solution.

### Cell viability assay

Cell viability was determined by MTT assay. Cells were seeded (2.5×10^3^ cells/well) into 96-well plate and treated with indicated concentrations of CDRI-85/287 for 48 h. At the end of incubation, MTT [3-(4, 5- dimethylthiazol-2-yl)-2, 5-diphenyl tetrazolium bromide] (0.5 mg/ml) (Sigma) was added and incubated for 2h at 37°C. After 2h of incubation, supernatants were removed and 100 µl of DMSO was added. The formazan crystals formed inside the viable cells were solubilized in DMSO and the OD was read with Microquant (Biotech, USA) at 540 nm. The IC_50_ value for the compound was determined by Compusyn software. The experiments were performed three times with five replicates in each.

### Co-immunoprecipitation assay

Interaction between EGF-EGFR proteins was studied by co-immunoprecipitating the complex followed by immunoblotting. Briefly, 2 µg anti-EGFR antibody was added to 500 µg of cell lysate and samples were incubated for overnight at 4°C with constant rocking. In negative control, cell lysate was incubated with corresponding non-immune serum instead of anti-EGFR. Following incubation, 100 µl of Protein A-Sepharose beads suspension was added and samples were incubated for 1 h at 4 °C. Immunoprecipitated complexes were collected by centrifugation at 3000×g for 2min at 4°C and washed three times with RIPA buffer. Immunoprecipitates were resuspended in Laemmli sample buffer to a final concentration of and heated for 5min at 95°C. The supernatants were collected by centrifugation at 12,000×g for 30 s at room temperature. Equal volume of immunoprecipitated proteins were run on 8% SDS-PAGE and transferred on PVDF membrane. The proteins were probed with anti-EGF, followed by the corresponding peroxidase conjugated secondary antibody. Bands were detected and analyzed by densitometry using Quantity One Software (v. 4.5.1) and a Gel Doc imaging system (Bio-Rad).

RETRACTED

### ELISA for EGFR activation

Levels of phosphorylated and total EGFR were quantified by using ELISA kit (Invitrogen). In brief, MDA-MB 231 or primary culture cells were treated as indicated in figure 2B. At the end of incubation, cell lysate was prepared by lysing the cells in buffer containing 10 mM Tris pH 7.4, 100 mM NaCl, 1 mM EDTA, 1 mM EGTA, 1 mMNaF, 20 mM Na4P2O7, 2 mMNa3VO4, 1%TritonX-100, 10% glycerol, 0.1% SDS and 0.5% deoxycholate supplemented with protease and phosphatase inhibitors. EGFR activation was measured by following the manufacturer’s instructions. OD was taken with Microquant ELISA reader (Biotech, USA) at 450 nm. The experiments were performed three times with three replicates in each.

**Figure 2:** CDRI-85/287 inhibits EGF- EGFR interaction and antagonizes EGF- induced EGFR activation. (A) Effect on EGF-EGFR complex formation as determined by co-immunoprecipitation in MDA-MB 231 cells. Cells were incubated as shown in the figure for 48 h. Cell lysates were immunoprecipitated with anti-EGFR antibody and subsequently immunoblotted with anti-EGF. NC is the negative control. Left panel shows the representative blot showing EGF-EGFR complex and right panel shows the densitometric analysis of bands. The results are presented as mean± SEM of three independent experiments. p values are a-p<0.001, b-p<0.01, c-p<0.05 and d-p>0.05 vs. control. (B, C) Effect of CDRI-85/287 on EGFR activation was determined by ELISA. Cells were treated as indicated in the figure and analyzed for the expression of phosphorylated EGFR and total EGFR using ELISA kit as per manufacturer’s instructions. Activation of EGFR at different concentrations (left panel) and at various time points (right panel) in (B) MDA-MB 231 and (C) primary breast adenocarcinoma cells was determined by normalizing the expression of p-EGFR with EGFR. p values are a-p<0.001, b<0.01, c-p<0.05 and d-p>0.05 vs. control.

RETRACTED

### Molecular Docking Analysis

The docking study was performed in AUTODOCK [25]. Prior to the docking, tyrphostin (AG-1478) and CDRI-85/287 were generated in SYBYL [26] and were subjected to optimization for their geometry using the Powell energy minimization algorithm, Gasteiger-Huckel charges, and 0.001 kcal/(mol.Å) as convergence criteria. The protein coordinates of EGFR from the EGFR - lapatinib (GW572016) co-crystal (PDB code: 1XKK) [27] were considered for investigating the binding modes of AG-1478 and CDRI-85/287. For docking study, the ligand-free protein was prepared in SYBYL by making use of the same procedure as adopted in case of study molecules. In SYBYL, using fit atom method, AG-1478 and CDRI-85/287 were positioned in 3D-space matching with lapatinib of co-crystal. The prepared EGFR protein and the corresponding study molecule were considered in AUTODOCK for the docking experiments. The grid size for the search of docking space was set at 60×60×60 distributed around the binding domain with a default grid spacing of 0.375 Å. The Lamarckian genetic algorithm was used for docking the molecules. For each molecule the docking was done with 100 runs. The molecules were allowed to flexibly dock into the protein coordinates (1XKK) to take their final conformation. The best docked conformers were collected from a population of 150 samples from 2.5 million energy evaluations. Along with AUTODOCK, Pymol [28] and MOE [29] software were used to visualize the interactions of protein and docked molecules. In order to validate the docking experiments lapatinib was also docked into the protein coordinates independent of its co-crystal structure. It has occupied almost the same position as that of lapatinib in co-crystal structure.

### Western blot analysis

CDRI-85/287 and vehicle treated cells and tumors from xenograft model were lysed in RIPA buffer (50 mM Tris pH-7.4, 150 mM NaCl, 1% nonidet-P40, 0.5% sodium deoxycholate, 0.1% SDS, 1 µM sodium orthovanadate) supplemented with protease inhibitor cocktail (Sigma) and 1 mM PMSF. Supernatant was collected by centrifugation at 13,000 rpm for 10 minutes. Equal amounts of protein were separated by gel electrophoresis and then transferred to Immuno-Blot™ PVDF membrane (Millipore). The membrane was blocked with 5% skimmed milk and then incubated with appropriate primary antibody overnight at 4 °C. The membrane was then washed and incubated with a secondary peroxidase conjugated antibody for 1 h. Antibody binding was detected using enhanced chemiluminescence detection system (GE Healthcare). After developing, the membrane was stripped and re-probed using another primary antibody of interest or β-actin to confirm equal loading. Each experiment was repeated three times to assess for consistency of results.

RETRACTED

Quantitation of band intensity was performed by densitometry using Quantity One® software (v.4.5.1) and a Gel Doc imaging system (Bio-Rad). Anti-PCNA, p-PI-3-K, PI-3-K, p-Akt, Akt, pNF-κB, NF-κB, p27, p-FOXO-3a, FOXO-3a, p-Rb, Rb, cyclin D1, EGF and anti- β-actin antibodies were purchased from Santa Cruz, CA, USA. Antibodies for EGFR, Bcl_2_, Bax, Bclxl, XIAP, p-MEK, MEK, p-Erk, Erk, c-fos, c-jun, cleaved caspase-3, -8, -9, and cleaved PARP were procured from Cell Signalling Technology, USA.

### Transient transfection and transactivation assay

MDA-MB 231 cells were seeded in 24 well plate and allowed to attain a confluency of 80–90%. Cells were then transfected with 100 ng of pAP1-Luc or p-c-fos-Luc or p-c-jun-Luc (Stratagene La Jolla, CA) using Lipofectamine -2000™ transfection reagent (Invitrogen) as per manufacturer’ protocol. To normalize for transfection efficiencies, 50 ng of pRL-SV40-luc (Promega, USA) was co-transfected. After 5 h of transfection, medium was changed and cells were treated with EGF, different concentrations of compound CDRI-85/287 or EGFR inhibitor, AG1478. After 18 h cells were lysed with passive lysis buffer. Luciferase activity was measured using Dual Luciferase Assay System (Promega) according to the manufacturer’s protocol to detect the transcriptional activity of the transfected promoter. The firefly luciferase intensity for each sample was normalized with transfection efficiency measured by renilla luciferase activity [30]. The experiments were performed three times with three replicates in each.

### Immunoflouresence imaging and confocal microscopy

Cells were grown on coverslips in 12-well plate and treated with vehicle, 3 and 7.5 µM of CDRI-85/287 in MDA-MB 231 and primary breast adenocarcinoma cells respectively for 24h. Cells were then fixed in methanol and acetone in 1∶1 ratio at 4°C and permeabilized with 0.1% Triton X-100. Cells were washed with PBS and blocked with 1% BSA and incubated with NF-κB antibody for overnight followed by 1h incubation with fluorescence-tagged secondary antibody, then counterstained with DAPI for 5 min. Images were captured at 63X using Carl Zeiss LSM 510 META microscope and analyzed using LSM Image Examiner Software to detect fluorescence and DAPI emissions.

RETRACTED

### Apoptosis analysis by flow cytometry

Human breast cancer MDA-MB 231 cells and primary breast cancer cells (2×10^5^ cells/ml) were cultured in 6-well plates and treated either with ethanol(vehicle) or with different concentrations of the compound. Adherent and detached cells were then harvested after 48 h, centrifuged and resuspended in 1 ml phosphate buffered saline (PBS). The Annexin V—FITC (fluorescein isothiocyanate)-labeled apoptosis detection kit (Sigma Chemical Co.) was used to detect and quantify apoptosis by flow cytometry as per manufacturer's instructions. Cells were analyzed using a flow cytometer (Becton Dickinson), and data were analyzed with CellQuest software.

### Cell cycle analysis by flow cytometry

Cells were seeded (2×10^5^cells/ml) in 6-well plates and treated with varying concentrations of CDRI-85/287 for 48h. After treatment, cells were washed with Phosphate buffered saline (PBS), fixed in 75% chilled ethanol, treated with RNase and then stained with propidium iodide (PI) (Sigma) solution (50 µg/ml). Cell cycle distribution was analyzed with fluorescence-activated cell sorter (Model FACS Calibur, BD biosciences, USA) and Cell- Quest software. The percentage of DNA content at different phases of the cell cycle was analyzed with Modfit-software (Verity Software House, ME, USA). The experiments were performed three times with three replicates in each.

### Caspase-3 colorimetric assay

Caspase-3 activity was measured using the colorimetric Caspase-3 assay kit (Sigma). Briefly, treated cells were trypsinized and centrifuged for 5min at 600 xg at 4°C. Then cell pellets were resuspended in ice-cold cell lysis buffer and incubated on ice for 20 min. At the end of the incubation, cell lysates were centrifuged at 20,000 x g for 10 min at 4°C. Supernatants were then incubated with 1 mM caspase-3 substrate (DEVD-pNA) for 2h at 37°C and the OD was measured at 405 nm. The experiments were performed three times with three replicates in each.

### Measurement of mitochondrial membrane potential (Δψm)

Δψm was estimated using JC-1 (cationic mitochondrial vital dye) as a probe using method as described previously [21]. Briefly, treated cells were collected and incubated for 20min with 5 µM JC-1 at 37°C, washed, and resuspended in media, and Δψm was measured at 590 nm for J-236 aggregates and at 530 nm for J-monomer. The ratio of 590/530 nm was considered as the relative Δψm value. The experiments were performed three times with three replicates in each.

### Transwell migration assay

Cell invasion assays were conducted in a 24-well format using matrigel-coated invasion chambers (BD Matrigel™Invasion Chambers; Cat # 354480) having a membrane pore size of 8.0 µm. Briefly, 2×10^5^ cells (MDA-MB-231) were seeded into the top chamber. The next day vehicle, EGF, 3 µM of compound, compound along with EGF and EGFR inhibitor was added into the bottom well for 12h. At the end of the treatment, the cells were post-stained with 0.1% crystal violet stain. The cells that invaded the BD Matrigel Matrix and passed through the pores of the BD FluoroBlok membrane were detected, photographed and counted under an inverted microscope (Nikon ECLIPSE TE2000-S, Nikon, Singapore).

RETRACTED

### Gelatin zymography

Zymography was performed in 10% polyacrylamide gels that had been cast in the presence of gelatin [15]. Briefly, samples (culture media) were resuspended in loading buffer and run on a 10% SDS-PAGE gel containing 0.5 mg/mL gelatin without prior denaturation. After electrophoresis, gels were washed to remove SDS and incubated for 30 min at room temperature in a renaturing buffer (50 mM Tris, 5 mM CaCl2, 0.02% NaN3, 1% Triton X-100). In the next step, gels were incubated for 48 h at 37°C in developing buffer [50 mM Tris-HCl (pH 7.8) 5 mM CaCl2, 0.15 M NaCl and 1% Triton X-100] and then subsequently stained with Coomassie Brilliant Blue G-250 and destained in 30% methanol, 10% acetic acid to detect gelatinase secretion.

### Tumour xenografts preparation in mice

All experimental procedures of this study were approved by Institutional Animal Ethics Committee (IAEC) of CDRI, Lucknow and IAEC of INMAS (DRDO), Delhi. Briefly, MDA-MB 231cells in normal saline were implanted subcutaneously into 6-week-old athymic nude mice bearing the nu/nu gene [NIH(s) (nu/nu)]. After the tumors attained the size of approx 2000 mm^3^, mice were treated with CDRI-85/287 (10 mg/kg body weight doses, per day for 16 days, p.o.) Animals of control group were treated with vehicle only. Xenograft tumor size was measured using Vernier callipers (major and minor axis) and tumor volume was calculated according to the equation: (L X W^2^)/2 (mm3), where L  =  length and W  =  width.

After euthanasia, animals were dissected for removal of tumors and various other organs for fixation in 4% formaldehyde for routine histology. Tissues were processed as per standard protocol.

### Statistical Analysis

Results are expressed as mean ±SEM for at least three separate determinations for each experiment. Statistical significance was determined by ANOVA and Newmann Keul’s test (for *in vitro*) or Student’s t-test (for *in vivo* studies). p values < 0.05 were considered significant.

## Results

### CDRI-85/287 strongly impaired the growth of EGFR over-expressing breast cancer cells and primary breast adenocarcinoma cells

CDRI-85/287 selectively inhibited the growth of estrogen receptor-negative and EGFR over-expressing MDA-MB 231 breast cancer cells while being non-toxic to normal human cells. (Fig. 1B). Treatment with the compound led to decrease in cell viability in a concentration dependent manner with IC_50_ of 3.7 µM in MDA-MB 231 cells (p<0.001). We also assessed the effect of compound on primary cells obtained from human breast carcinoma over-expressing EGFR. The compound inhibited the growth of these cells with IC_50_ of 7.9 µM (Fig. 1B). The compound was also found to significantly inhibit EGF-induced proliferation (p<0.001vs. EGF at 1 µM in MDA-MB 231 and p<0.01 vs. EGF at 2.5 µM in primary breast cancer cells) suggesting that it acts by antagonising EGF action in inhibiting proliferation of these cells.

RETRACTED

In normal kidney cell lines HEK-293 and VERO cells, the compound treatment did not cause significant inhibition of cell viability, upto 40 µM concentration (Fig. S1).

### CDRI-85/287 inhibits EGF- EGFR interaction and antagonises EGF- induced EGFR activation

To identify the molecular characteristics responsible for compound’s toxicity, we sought to investigate the diverse biological responses triggered in ER-ve breast cancer cell lines by the compound. Since the compound was found to inhibit EGF- induced proliferation of breast cancer cells, we went onto see if the compound also prevents binding of EGF to EGFR. Co-immunoprecipitation studies indicated that CDRI-85/287 like AG1478 significantly reduced the formation of EGF-EGFR complex both per se (p<0.01) and in presence of EGF (p<0.01) (Fig. 2A).

Further, we analyzed the effect of compound on EGFR activation using ELISA (Fig. 2B,C). After 30 min of incubation, the compound significantly decreased phospho form of EGFR which further decreased with time upto 3 h in both MDA-MB 231 cells(p<0.05 to p<0.001) and primary breast adenocarcinoma cells (p<0.01 to p<0.001) while 100 ng/ml of EGF induced tyrosine phosphorylation of EGFR (p<0.01). In a dose-dependent study, the compound inhibited both basal as well as EGF-induced activation of EGFR. At 2 µM concentration, the compound significantly inhibited (p<0.05) the phosphorylation of EGFR and the decrease was more significant at 3 µM (p<0.01) in presence of EGF in case of MDA-MB 231 cells. In primary breast cancer cells, significant inhibition of EGFR activation was observed at 5 µM (p<0.01) both in absence and in presence of EGF. Significant change in the level of total EGFR was not observed in the two cell lines on treatment with indicated concentrations of the compound.

### CDRI-85/287 displays a higher binding affinity for EGFR than AG1478

The docking experiments indicate that AG-1478 and CDRI-85/287 occupy a position in ATP-binding pocket of EGFR which is comparable to that of lapatinib. In the binding pocket, the quinazolin moiety of lapatinib occupied the central place with benzyloxyphenyl and furan-methylamine moieties extending to its (quinazolin) either side (binding energy -11.61 Kcal/mol) (Fig. 3A). However, in the binding pocket, AG-1478 has shown only partial occupancy (binding energy: −8.47 Kcal/mol; IC_50_ = 10 µM). The docking poses have indicated that the AG-1478’s quinazolin and 3-chloro aniline moieties have respectively occupied the positions of quinazolin and benzyloxyphenyl moieties of lapatinib. AG-1478 has no structural moiety to satisfy the space corresponding to furan-methylamine moiety of lapatinib (Fig. 3B). This may be a reason for AG-1478’s weak binding to EGFR. Interestingly the docking pose as well as binding pocket occupancy of CDRI-85/287 is comparable to that of lapatinib (binding energy: -10.01 Kcal/mol; IC_50_ = 2.5 µM) (Fig. 3C). Here the chroman and N-ethyl-piperidinyl moieties of CDRI-85/287 have occupied the binding areas of benzyloxyphenyl and furan-methylamine moieties of lapatinib, respectively. The aryl-bridge between the chroman and N-ethyl-piperidinyl moieties of CDRI-85/287 has served the purpose of quinazolin moiety of lapatinib. The differences in the binding energy of AG-1478 and CDRI-85/287 to EGFR have corroborated their activity.

RETRACTED

**Figure 3:** Molecular Docking analysis of CDRI-85/287 with EGFR. (A) Schematic partitioning of Lapatinib in the ATP-binding pocket. In the binding pocket quinazolin moiety of lapatinib has occupied the central place with benzyloxyphenyl and furan-methylamine moieties extending to its either side (wing I & II respectively). (B) Schematic partitioning of AG 1478 in the ATP-binding pocket. The chlorobenzene moiety of AG 1478 are designated as wing-I & dimethoxy moiety partially represent wing II site. The quinazoline moiety of AG 1478 has acted as central part of the scaffold. (C) Comparison of CDRI 85/287 structural moieties with AG 1478. (D) Docked conformation of AG 1478 with wild type EGFR protein (PDB ID. 1XKK). Red dash indicate H-bond interaction site with of EGFR where cyan, magenta & salmon colour specify alpha-helix, beta-sheet & loop regions of protein correspondingly. (E) Docked conformation of CDRI 85/287 analogue with EGFR protein (PDB ID 1XKK). Red dash shows H-bond interaction site with same protein site. (F) Superimposition of AG 1478 & CDRI 85/287 in a same protein binding pocket shows H-bond interaction with ASP855 & MET793 residues respectively. (G) Superimposition of Lapatinib (magenta), AG 1478 (green) and CDRI 85/287 derivative (Cyan). (H) Schematic 2D-representation of AG 1478. (I) proposed binding mode of CDRI 85/287 analogue with surrounding residues in the ATP-binding pocket of EGFR.

RETRACTED

### CDRI-85/287 interferes with MEK/Erk activation and downstream signaling

Next, we sought to study the effect of compound on MEK/Erk pathway involved in cell proliferation and invasion. In MDA-MB 231 cells, EGF significantly induced the activation of MEK which in turn led to activation of downstream MAPK, Erk (Fig. 4A). The compound at 3 µM significantly led to inhibition of MEK (p<0.001vs. control) and Erk (p<0.05vs. control) activation as evidenced by decreased expression of phospho forms of the proteins. Likewise, in primary breast adenocarcinoma cells the compound interfered with Erk activation leading to decreased levels of p-Erk (p<0.05 vs control) both in presence and in absence of EGF (Fig. 4A).

**Figure 4:** CDRI-85/287 interferes with MEK/Erk activation to inhibit downstream signaling. (A) Western blot analysis to see the expression of p-MEK, MEK, p-Erk and Erk. MDA-MB 231 (left panel) and primary breast cancer cells (right panel) were treated with the indicated concentrations of CDRI-85/287 for 24h and 30 µg of whole cell lysate in each lane was probed for the expression of different proteins using specific antibodies. Representative blots are shown in the upper panel and densitometric quantitation of protein expression levels are shown as fold changes in the lower panel. Results are expressed as mean ± SEM, n = 3. p values are a-p<0.001, b<0.01, c-p<0.05 and d-p>0.05 vs. control. (B) Transcriptional activation of the AP-1 promoter complex in transiently transfected MDA-MB 231 cells in response to CDRI-85/287 alone or in the presence of 100 ng/ml EGF. MDA-MB 231 cells were transfected with pAP1-Luc or p-c-fos-Luc or p-c-jun-Luc reporter plasmids and incubated with various concentrations of compound for 24h. pRL-luc plasmid was used as internal control. Results are described as % of normalized relative luciferase unit (RLU). Results are expressed as mean ± SEM, n = 3. p values are a-p<0.001, b-p<0.01, c-p<0.05 and d-p>0.05 vs. control and e-p<0.001, f-p<0.01, g-p<0.05 and h-p>0.05 vs. EGF. (C) Effect of compound on AP-1 dependent proliferation markers. MDA-MB 231 (left panel) and primary breast cancer cells (right panel) were treated with the indicated concentrations of compound for 48h. 30 µg of whole cell lysate in each lane was probed for the expression of different proteins using specific antibodies. Representative blots are shown in the upper panel and densitometric quantitation of protein expression levels are shown as fold changes in the lower panel. Results are expressed as mean ± SEM, n = 3. p values are a-p<0.001, b<0.01, c-p<0.05 and d-p>0.05 vs. control.

RETRACTED

Since Erk exerts part of its proliferative activity via AP-1 transcriptional complex, we next studied the effect on AP-1 transcriptional complex. For this we analyzed AP-1 transcriptional activation in MDA-MB 231 cells transiently transfected with AP-1 reporter plasmid. EGF increased the promoter activity of AP-1 transcriptional complex while the compound inhibited AP-1 promoter activity (Fig. 4B). The compound also inhibited the transcriptional activity of c-fos and c-jun, components of AP-1 transcriptional assembly in MDA-MB 231 cells transiently transfected with the respective reporter constructs. The compound also inhibited EGF induced transcriptional activation of AP-1 transcriptional machinery. AG1478 decreased the transcriptional activation via AP-1 complex since it blocks EGFR activation upstream. The compound also significantly reduced the levels of AP-1 dependent proliferation markers including PCNA, IGF-1, c-fos and c-jun in both MDA-MB 231 cells and primary breast adenocarcinoma cells (Fig. 4C).

### Modulation of PI-3-K/Akt, NF-κB and FOXO signaling and downstream effectors

We further analyzed several major components of signaling pathways downstream of EGFR. We analyzed the effect of the compound on activation of PI-3-K and its downstream Akt. EGF significantly induced phosphorylation of PI-3-K which in turn increased phosphorylation of Akt (p<0.01vs.control) while the compound decreased the phosphorylated forms of the proteins, PI-3-K (p<0.01) and Akt (P<0.05). The compound significantly decreased the phosphorylation of the proteins even in the presence of EGF (p<0.05 vs control) thus showing that the compound acts by antagonizing EGF in deactivating these proteins and preventing further downstream signaling in both MDA-MB 231 and primary breast cancer cells (Fig. 5). The next objective was to study the effect of compound on NF-κB activation. The compound significantly reduced the phosphorylated form of NF-κB protein as evidenced by western blotting. Another downstream target of Akt is the Forkhead transcription factor FOXO-3a, which in its active form leads to transcription of genes involved in cell cycle arrest and prevents cellular proliferation [13]. The compound CDRI-85/287 decreased the expression of phosphorylated FOXO-3a in both MDA-MB 231 and primary breast cancer cells in contrast to EGF which in turn prevented its proteasomal degradation leading to increased expression of FOXO-3a protein confirmed by immunoblotting studies (Fig. 5). This unphosphorylated FOXO-3a remains in active form and would lead to modulation of cell cycle regulatory genes.

RETRACTED

**Figure 5:** CDRI-85/287 modulates PI-3-K/Akt, NF-κB and FOXO-3a pathway. Analysis of PI-3-K, Akt, NF-kB and FOXO phosphorylation in (A) MDA-MB 231 and (B) primary breast adenocarcinoma cells. Cells were treated with the indicated concentrations of compound for 24h and 30 µg whole cell lysate in each lane was probed for the expression of different proteins using specific antibodies. β-actin was used as a control to correct for loading. Representative blots are shown in left panel and densitometric analysis of bands is shown in right panel. Results are expressed as mean ± SEM, n = 3. p values are a-p<0.001, b<0.01, c-p<0.05 and d-p>0.05 vs. control.

Next, we analyzed the localization pattern of NF-κB under the effect of compound. Immunoblotting experiment displayed that the compound decreased both basal as well as EGF-induced expression of nuclear NF-κB while increased expression in cytosolic fraction (Fig. 6A). These results were validated by confocal microscopy that clearly indicates that 3 µM of CDRI-85/287 significantly decreased the nuclear pool of NF-κB protein (Fig. 6B).

**Figure 6:** Effect of compound on downstream effectors of NF-κB and FOXO-3a. (A) Western blot analysis to see the nuclear and cytosolic expression of NF-κB in MDA-MB 231 cells. Cells were treated as shown in the figure for 48h. Nuclear and cytosolic proteins were extracted following manufacturer’s instructions and subjected for immunoblotting using anti-NF-κB antibody. Representative blots are shown in the left panel and densitometric quantitation of protein expression levels are shown as fold changes in the right panel. Results are expressed as mean ± SEM, n = 3. p values are a-p<0.001, b<0.01, c-p<0.05 and d-p>0.05 vs. control. (B) Confocal microscopy to demonstrate the effect of compound on localization pattern of NFκB (p65). MDA-MB 231 and primary breast cancer cells were treated with vehicle or indicated concentration of compound for 24 hrs. Cells were fixed, permeabilized, incubated with NFκB antibody for overnight, and incubated with FITC-conjugated anti-rabbit antibody for 1 h. The preparations were washed and counterstained with DAPI and images were captured at 63X using Carl Zeiss LSM 510 META microscope. Representative micrographs demonstrating the subcellular distribution of NFκB are shown. (C) Transcriptional activation of the NF-κB promoter in transiently transfected MDA-MB 231 cells in response to compound either alone or in the presence of 100 ng/ml EGF. MDA-MB 231 cells were transfected with pNF-κB-Luc reporter plasmids and incubated with various concentrations of CDRI-85/287 for 24h. pRL-luc plasmid was used as internal control. Results are described as % of normalized relative luciferase unit (RLU). Results are expressed as mean ± SEM, n = 3. p values are a-p<0.001, b-p<0.01, c-p<0.05 and d-p>0.05 vs. control and e-p<0.001, f-p<0.01, g-p<0.05 and h-p>0.05 vs. EGF. (D) Western blot analysis for the expression of cell cycle regulatory and anti-apoptotic proteins (Bclxl and XIAP) in MDA-MB 231 (left panel) and primary breast cancer cells (right panel). Cells were treated with the indicated concentrations of compound for 48h and 30 µg whole cell lysate in each lane was probed for the expression of different proteins using specific antibodies. β-actin was used as a control to correct for loading. Representative blots are shown. Densitometric analysis of bands is shown in Fig. S2.

RETRACTED

Further, the basal as well as EGF-induced promoter activity of NF-κB determined by transient transfection and transactivation assay in MDA-MB 231 cells was also found to decrease with increasing concentrations of the compound (p<0.001) (Fig. 6C).

Next, we observed the effect of compound on downstream effectors of NF-κB and FOXO-3a. The compound led to increase in the expression of cell cycle dependent kinase inhibitor p27 in both MDA-MB231 and primary breast cancer cells (Fig. 6D). Increased levels of p27 led to decrease in the expression of cyclin D1 by the compound which in turn prevented phosphorylation of Rb protein maintaining it in unphosphorylated state as evidenced by the expression of total Rb. Unphosphorylated Rb sequesters and inactivates E2F preventing cell cycle progression from G1 to S phase by inhibiting the transcription of E2F dependent genes. CDRI-85/287 also decreased the expression of Bclxl and XIAP, the anti-apoptotic members of Bcl_2_ family. The results suggest that the compound exerts its effect via modulation of cell cycle progression and apoptosis induction.

### CDRI-85/287 caused G1/S phase arrest in EGFR-overexpressing breast cancer cells

We next studied the effect of CDRI-85/287 on cellular distribution at different stages of the cell cycle in breast cancer cells. For this, flow cytometric analysis of PI-stained cells was done. CDRI-85/287 led to increased accumulation of cells in G1 phase of the cycle in both MDA-MB 231 and primary breast cancer cells (p<0.01 at 3 µM and 7.5 µM in MDA-MB 231 and primary breast cancer cells respectively), delaying progression into synthesis phase (Fig. 7A). G1/S phase arrest was further confirmed by studying the expression of cyclins, cdks and CKIs. The compound significantly reduced the expression of cyclin D1, cyclin E1, cdk4 and increased the expression of cell cycle inhibitory proteins p21 and p27 in a concentration dependent manner in MDA-MB231 cells (Fig. 7B). However, the expression of cyclin A1 was not significantly altered by the compound. The results clearly indicated that CDRI-85/287 inhibits growth of ER-negative breast cancer cells by inhibiting cell cycle progression from G1 to S phase.

RETRACTED

**Figure 7:** Inhibition of cell cycle progression by CDRI-85/287. (A) Cell cycle analysis by flow cytometry. MDA-MB 231 and primary breast cancer cells were treated with the indicated concentrations of compound for 48h. The cells stained with propidium iodide (PI) were subjected to flow cytometric analysis to determine the percentage of cells at each phase of the cell cycle. Representative images of flow cytometry of vehicle and compound treated cells are shown in the upper panel and the percentage of cell with SEM based on three independent experiments is shown in the lower panel. p values are a-p<0.001, b<0.01, c-p<0.05 and d-p>0.05 vs. control. (B) Western blot analysis to see the expression of cell cycle regulatory proteins cyclin D1, A1, B1, cdk4, p21 and p27. MDA-MB 231 and primary breast cancer cells were treated with the indicated concentrations of compound for 48h and 30 µg whole cell lysate in each lane was probed for the expression of different proteins using specific antibodies. β-actin was used as a control to correct for loading. Representative blots are shown in the upper panel and densitometric quantitation of protein expression levels are shown as fold changes in the lower panel. Results are expressed as mean ± SEM, n = 3. p values are a-p<0.001, b<0.01, c-p<0.05 and d-p>0.05 vs. control.

### CDRI-85/287 induced apoptosis in MDA-MB 231and primary breast adenocarcinoma cells via mitochondrial pathway

Decrease in the expression of anti-apoptotic proteins XIAP and Bclxl prompted us to check if the loss in cell viability on treatment with the compound is due to induction of apoptosis. For this we did flow cytometric analysis of Annexin V/PI stained cell treated with vehicle or different concentration of the compound. The compound significantly increased the percentage of apoptotic cells in a concentration-dependent manner, and more than 50% of the cells displayed apoptosis at 5 µM in MDA-MB 231(p<0.001) and at 7.5 µM in primary breast cancer cells (p<0.001) corresponding with the results of cell proliferation assay (Fig. 8A).

**Figure 8:** Analysis of apoptosis in MDA-MB 231 and primary breast adenocarcinoma cells. (A) Cells treated with vehicle and CDRI-85/287 were analyzed by flow cytometry of annexin-V/PI stained cells after 48h culture. AV^+^/PI^−^ - intact cells; AV^−^/PI^+^ -nonviable/necrotic cells; AV^+^/PI^−^ and AV^+^/PI^+^ - apoptotic cells. Representative images are shown in the upper panel and the percentage of cell fraction with SEM based on three independent experiments is shown in the lower panel. p values are a-p<0.001, b-p<0.01, c-p<0.05 and d-p>0.05 vs. control. (B) Western blot analysis to see the expression of pro- and anti- apoptotic proteins. MDA-MB 231 and primary breast cancer cells were treated with the indicated concentrations of compound for 48h, and 30 µg whole cell lysate in each lane was probed for the expression of different proteins using specific antibodies. β-actin was used as a control to correct for loading. Representative blots are shown in the upper panel and densitometric quantitation of protein expression levels are shown as fold changes in the lower panel. Results are expressed as mean ± SEM, n = 3. p values are a-p<0.001, b<0.01, c-p<0.05 and d-p>0.05 vs. control.

RETRACTED

Apoptosis was also evident upon examination of caspase-3 activity in MDA-MB 231 cells which was determined by incubating the cellular extracts with caspase-3 substrate (DEVD-pNA). Caspase 3 activity was significantly up-regulated by 1.5- fold and 2.5-fold in MDA-MB 231 cells that were treated with 2 and 3 µM of CDRI-85/287 respectively (p<0.05 at 1 µM to p<0.001 at 3 µM) (Fig. S3A). However in presence of caspase-3 inhibitor, no change in caspase-3 activity was observed on treatment with the compound. These results indicated that compound exerts its anti-proliferation activity in tumor cell-specific manner by activating the caspase pathway followed by induction of apoptosis. Further we went on to explore the pathway involved in execution of apoptosis. Alterations in the mitochondrial transmembrane potential (ψ_m_) has been shown to be important for the release of mitochondrial proteins such as cytochrome c, which when in the cytosol can lead to activation of the caspase cascade and subsequent death [31]. Therefore, we measured Δψ_m_ using the JC-1 dye and the results showed a significant drop (p<0.001) in Δψ_m_ in the presence of 3 µM of CDRI-85/287 in MDA-MB 231 and at 7.5 µM in primary cancer cells (Fig. S3B). These results indicate that the apoptotic-signaling pathway activated by compound is likely to be mediated via the mitochondrial pathway.

Next, we evaluated the levels of the pro- and anti-apoptotic proteins. While the level of Bax increased at protein level (Fig. 8B), compound triggered a dose-dependent decrease in the levels of anti-apoptotic Bcl_2_ in both cancer cell lines. CDRI-85/287 elicited a dose-dependent increase in the Bax/Bcl_2_ ratio, reaching upto 15-fold (p<0.001) and 9-fold (p<0.001) at IC_50_ concentration in MDA-MB231 and primary cancer cells respectively, thus mediating induction of apoptosis via intrinsic pathway. To further elucidate the role of CDRI-85/287 in inducing apoptosis, cells were treated with indicated concentrations of the compound and the whole cell lysates were probed for the expression of cleaved caspase-8, -9, -3 and cleaved PARP. Compound treatment caused a dose-dependent increase in the level of cleaved caspase-9, -3 and cleaved PARP in MDA-MB 231 and primary cancer cells. The expression of cleaved caspase-8 was not observed excluding the possibility of involvement of extrinsic pathway in the action of compound.

RETRACTED

### Inhibition of EGF-induced MDA-MB 231 cell invasion by CDRI-85/287

We next studied the effect of compound on EGF-induced invasion of MDA-MB 231 (Fig. 9A). We found that EGF significantly increased the invasion of MDA-MB 231 cells (p<0.001). The level of EGF-induced cell invasion was 157% of control group. However, both basal as well as EGF- induced cell invasion were suppressed by treatment with 3 µM of CDRI-85/287 (p<0.01). EGF-induced cell invasion was decreased by 72% of control level in response to 3 µM of compound.

**Figure 9:** Effect of compound CDRI-85/287 on the invasive properties of MDA-MB 231 cells. (A) Transwell migration assay. MDA-MB231 cells were seeded in the upper chamber with vehicle, EGF, CDRI-85/287, EGF along with the compound CDRI-85/287 or AG1478 added in the lower chamber. Cells that migrated to the low chamber were fixed, stained, and counted by light microscopy as described in Methods (left). These results are representative images of three independent experiments. The graph in the right panel shows the average number of migrated cells in three wells from three independent experiments (random fields were scanned and number of cells from four fields per well were counted). Results are expressed as mean ± SEM, n = 3. p values are a-p<0.001, b<0.01, c-p<0.05 and d-p>0.05 vs. control. (B) Inhibition of MMP-9 activity by CDRI-85/287 in breast cancer cells. MDA-MB 231 cells were treated as indicated for 12 h, conditioned media was collected and MMP activity was analyzed by gelatin zymography. Upper panel shows the representative gel image and lower panel shows the densitomentric analysis of band intensity. Results are expressed as mean ± SEM, n = 3. p values are a-p<0.001, b<0.01, c-p<0.05 and d-p>0.05 vs. control. (C) Western blot analysis to demonstrate the effect of CDRI-85/287 on the expression of CTGF in conditioned media. Cells were treated with increasing concentrations of CDRI-85/287 for 24 h, conditioned media was collected and subjected to western blotting for the expression of CTGF. Results are expressed as mean ± SEM, n = 3. p values are a-p<0.001, b<0.01, c-p<0.05 and d-p>0.05 vs. control

Next, we investigated if the compound suppresses MMP-9 activity in MDA-MB 231. MMP-9 (92 kDa gelatinase) is particularly known to play a critical role in cancer progression, such as angiogenesis as well as tumor growth, invasion and distant metastasis of various tumors and breast cancer as well [10], [15]. We found that EGF induced MMP-9 activity (p<0.05) while the compound decreased it significantly both in absence and in presence of EGF (p<0.001 and p<0.01 respectively in comparison to the control group) (Fig 9B).

RETRACTED

We also analyzed the expression of CTGF in conditioned media of MDA-MB 231 cells and found a concentration dependent decrease in the expression of CTGF secreted by these cells (p<0.05 to p<0.01 vs. control). Therefore, we demonstrated that CDRI-85/287 suppresses EGF-induced cell invasion through inhibition of MMP-9 activity and CTGF expression in MDA-MB 231 cells (Fig 9C).

### Benzopyran derivative CDRI-85/287 suppresses the growth of tumor xenograft in nude mice

In vivo studies demonstrated that the compound at 10 mg/kg body weight/day significantly reduced tumor volume in xenograft mice model (Fig. 10A). The average tumor size in this group was 66% lower after 16 days of treatment compared with vehicle treated group (Fig. 10C). Histological assessment showed that tumors from vehicle-treated mice were primarily composed of tumor epithelial cells with small amounts of mouse-derived stroma and frequent blood vessels. Tumors from mice treated with CDRI-85/287 presented with large areas of stroma where deletion of epithelial cells had occurred. Cellular apoptosis was also evident in compound treated group (Fig. 10B) in comparison to the tumor from the vehicle treated group. Significant change was not observed in body weight in the vehicle and treated group (Fig 10D).

**Figure 10:** Effect of CDRI-85/287 on tumor regression in MDA-MB 231 xenograft mouse model. (A) Representative images of MDA-MB 231 xenograft nude mice showing regression in tumor volume after treatment with CDRI-85/287(10 mg/kg, p.o.) in comparison to vehicle treated (VT) group. (B) Upper panel shows the dissected out tumors from vehicle treated and CDRI-85/287 treated xenograft mice. Lower panel shows representative images of hematoxylin and eosin stained tissue sections from vehicle- and CDRI-85/287 treated groups. (C) Graph showing tumor volume changes within 16 days after initiation of treatment (marked by arrow). Number of animals per group  =  6 to 8. (D) The average body weights of the mice during tumor development and treatment (marked by arrow). Number of animals per group  =  6 to 8.

Histomorphology did not show any marked change in liver, lungs, spleen, uterus and kidney of the compound treated mice as compared to vehicle treated control group (Fig. S4).

RETRACTED

### CDRI-85/287 inhibits EGFR activation, MEK/Erk and PI-3-K/Akt pathway in xenograft tissue

Treatment with the compound led to significant reduction in phosphorylated forms of EGFR (p<0.001) and Erk (p<0.01) in comparison to vehicle treated group. A significant decrease was also observed in the expression of PCNA (p<0.01), c-fos (p<0.05), c-jun (p<0.01)and IGF-1(p<0.01) in compound treated group in comparison to vehicle treated mice (Fig. 11A).

**Figure 11:** Effect of CDRI-85/287 on EGFR pathway in xenograft tissue. Western blot analysis to determine the effect of CDRI-85/287 on (A) activation of EGFR and MEK/Erk pathway, (B) activation of PI-3-K/Akt and expression of downstream effectors, and (C) the expression of pro- and anti- apoptotic proteins in vehicle and CDRI-85/287 treated xenograft tissue. 30 µg whole cell lysate in each lane was probed for the expression of different proteins using specific antibodies. β-actin was used as a control to correct for loading. Representative blots are shown in the left panel and densitometric quantitation of protein expression levels are shown as fold changes in the right panel. Results are expressed as mean ± SEM, n = 3. p values are a-p<0.001, b<0.01, c-p<0.05 and d-p>0.05 vs. control.

Western blot analysis indicated that the compound led to a decrease in the phosphorylated forms of Akt, NF-κB and FOXO-3a leading to decreased activation of NF-κB and increased activation of FOXO-3a in tumors from CDRI-85/287 treated xenograft mice in comparison to vehicle treated group. This in turn resulted in increased levels of p27 and decreased levels of cyclin D1, phosphorylated Rb and decreased expression of total Rb in compound treated xenograft tumor (Fig. 11B).

Further, significant decrease was observed in the expression of anti-apoptotic protein Bclxl, XIAP and Bcl_2_ whereas the expression of Bax, cleaved caspase-9, cleaved caspase-3 and cleaved PARP was increased in compound treated mice (Fig. 11C). These results showed that compound caused the induction of apoptosis via intrinsic pathway and reduced the tumor growth.

## Discussion

In search for novel agents for successful therapies of breast cancer, EGFR has long been used as a target for therapeutic intervention in ER-ve as well as triple negative breast tumors that do not respond to endocrine therapy [1]. In the present study, we have examined the effects of 2-[piperidinoethoxyphenyl] -3- phenyl- 2H-benzo (b) pyran (CDRI-85/287) on EGFR -mediated signaling and cell survival/apoptosis in ER- negative human breast cancer cells and in xenograft mice model. Initial findings suggest that CDRI-85/287 showed cytotoxic effects in ER- negative breast cancer cells MDA-MB231 and in human primary culture and caused regression in tumor size in MDA-MB 231 xenograft in mice.

RETRACTED

While exploring the mechanistic action of compound, we found that the compound exerts anti-proliferative and anti-invasive activity via interfering with EGF binding to EGFR and inhibition EGFR activation as observed in MDA-MB 231 and primary breast cancer cells. Docking studies revealed that CDRI-85/287 displayed better binding affinity to EGFR in comparison to the EGFR inhibitor AG1478. It has also been demonstrated by several investigators that transient activation of ERK1/2, a downstream effector of EGFR, also plays a pivotal role in cellular proliferation and leads to cell cycle arrest and causes induction of apoptosis [32]. The MEK/Erk pathway exerts its growth promoting effects via AP-1 transcriptional complex. Thus inhibition of Erk activation caused by the compound led to inhibition of activation of AP-1 transcriptional complex as evidenced by decrease in the EGF -induced transcriptional activation via AP-1, c-fos and c-jun. This in turn led to decreased expression of proliferation markers and prevented growth of breast cancer cells. These findings co-related well with the results obtained from *in vivo* studies in MDA-MB 231 tumor xenograft where anti-tumor response was observed in 85/287- treated mice.

The mitogenic effect of EGF is also mediated via activation of PI-3-kinase and IκK-dependent activation of NF-κB and inhibition of FOXO activity [12]–[14]. Our results indicated that the compound CDRI-85/287 inhibited the activation of PI-3-K and Akt which led to inhibition of activation of downstream effector NF-κB and enhanced activation of FOXO-3a. The transcription factor NF-κB is well established as a regulator of genes encoding cytokines, cytokine receptors, and cell adhesion molecules that drive immune and inflammatory responses. It can regulate genes involved in both proliferation and apoptosis including anti-apoptotic genes BclxL and XIAP and growth inducible ErbB2 and cyclin D1 [33]. On the other hand FOXO-3a is known to suppress the activity of NF-κB by inducing IκB-Ras1 [34]. Upon treatment with our compound, the activation of FOXO-3a further led to increased expression of p27^kip^, cyclin dependent kinase inhibitor and decreased expression of cyclin D1. Decreased cyclin D1 expression led to decreased phosphorylation of tumor suppressor Rb protein thus maintaining it in active state. Active Rb sequesters E2F preventing transcription of genes involved in cell cycle progression from G1 to S phase. This was confirmed by concentration dependent decrease in the expression of cyclin E1, A1, D1, cdk4 and increased expression of cell cycle inhibitory proteins p21 and p27.

RETRACTED

The decreased activity of NF-κB and increased activity of FOXO-3a led to decrease in the expression of anti-apoptotic proteins Bclxl and XIAP both *in vitro* and *in vivo* leading to induction of apoptosis as evidenced by flow cytometry in MDA-MB 231 and primary breast adenocarcinoma cells. Further, the compound led to decreased Bax: Bcl_2_ ratio which might be responsible for significant decrease in mitochondrial membrane potential as observed with compound treatment. The reduced expression of Bcl_2_ and the presence of cleaved fragments of caspases-9,-3 and PARP in treated cells and in xenograft tumors confirmed the involvement of mitochondrial pathway of apoptosis triggered by these compounds. The expression of cleaved caspase-8 was not detectable which confirmed that caspase-8 pathway does not participate in CDRI-85/287 induced apoptosis in ER- negative MDA-MB 231 cells and primary breast cancer cells (data not shown). Finally, CDRI-85/287 arrested tumor growth in a MDA-MB 231 xenograft model of human estrogen receptor-negative breast cancer, showing that the potent effect of this compound could also be manifested in vivo, with concomitant inhibition of EGFR pathway in the treated tumors.

It is reported that PI-3-K pathway and MAP kinase pathway are also involved in the EGFR-mediated modulation of cell invasion [35], [36]. Tumor cell migration and invasion is a critical factor for malignant tumor metastasis, which is a multiple process that requires the degradation of the extracellular matrix both at the primary tumor site and at the secondary colonization site. This degradation process is dependent on the activity of specific endopeptidases, the matrix metalloproteinases (MMPs). MMP-9 expression has been related to the invasive property of a variety of cancers including breast carcinoma [15]. MDA-MB 231 is a highly metastatic breast cancer cell line and expresses high level of MMP-9. Our data showed that compound prevented invasion of MDA-MB 231 cells via matrigel membrane and also significantly suppressed the MMP-9 activity in MDA-MB 231 cells. The expression of connective tissue growth factor, CTGF which again is an indicator of the invasive properties of the cell [37] was found to decrease in conditioned media on treatment with the compound. Connective tissue growth factor (CTGF) expression is elevated in advanced stages of breast cancer, and the regulatory role of CTGF in invasive breast cancer cell phenotypes has already been reported [38].

In conclusion, the present study demonstrates the anti-proliferative and anti-tumorigenic effect of CDRI-85/287 in ER-negative breast cancer cells and in xenograft mouse model, respectively. The study provides evidence that CDRI-85/287 exerts its anti-proliferative and anti-invasive properties via preventing EGFR activation and subsequently inhibits the tumor growth by inhibiting PI-3-K/Akt and MEK/Erk pathways. Inhibition of cell invasion through matrigel membrane and reduced MMP-9 activity confirms that apart from anti-proliferative properties, compound can efficiently block EGF- stimulated invasion of breast cancer cells. Based on these observations, we have hypothesised the working model of CDRI-85/287 as an anti-cancer agent in ER-negative tumors (Fig 12). In total, our observations strongly suggest that benzopyran derivative CDRI-85/287, due to its anti-proliferative and anti-invasive properties, can be rated as a promising candidate for future development as a novel therapeutic treatment strategy for more aggressive forms of breast cancer. In addition, such compounds may be effective in blocking the growth factor – mediated signaling in cases where resistance to endocrine therapy has occurred, although this needs to be proven under specific experimental conditions.

RETRACTED

**Figure 12:** Schematic representation of the action of compound on inhibition of EGFR signaling. The compound competes with EGF in activating EGFR and leads to subsequent induction of apoptosis, inhibition of cell cycle progression and cell invasion.

## Supporting Information

Figure S1 **Cytotoxicity of CDRI-85/287 in non-cancerous cells determined by MTT assay.** Values are mean± SEM, n = 5; p value: d- p>0.05 (insignificant).
(TIF)

Figure S2 **Effect of compound on the expression of downstream effectors of NF-κB and FOXO-3a.** Densitometric analysis of the western blots showing effect of compound on the expression of p27, cyclin D1, p-Rb/Rb, XIAP and Bclxl in MDA-MB 231(left panel) and primary breast adenocarcinoma cells (right panel). Results are expressed as mean ± SEM, n = 5. p values are a-p<0.001, b<0.01, c-p<0.05 and d-p>0.05 vs. control.
(TIF)

Figure S3 **CDRI-85/287 induces apoptosis via intrinsic pathway in breast cancer cells.** (A) Induction of caspase-3 proteolytic activity in MDA-MB 231 cells treated with CDRI-85/287 for 48 h. Proteolytic activity was measured by cleavage of the caspase-3 substrate DEVD-pNA. Results are expressed as mean ± SEM, n = 5. p values are a-p<0.001, b<0.01, c-p<0.05 and d-p>0.05 vs. control. (B) MDA-MB 231 and primary breast cancer cells were treated with 3 and 7.5 µM of CDRI-85/287 for 24h. Mitochondrial membrane potential was measured by normalization of the 590:530 nm JC-1 emission ratios and then normalized to untreated cells. Results are expressed as mean ± SEM, n = 3. a-p<0.001 vs. control.
(TIF)

Figure S4 **Representative sections of kidney, liver, lung, spleen and uterus of vehicle treated and CDRI-85/287 treated mice.** Photomicrographs of histological sections were captured. Number of animals per group = 6 to 8.
(TIF)

RETRACTED

## References

[1] SaxenaR, DwivediA (2012) ErbB family receptor inhibitors as therapeutic agents in breast cancer: current status and future clinical perspective. Med Res Rev 32 (1): 166–215.2218379710.1002/med.20209

[2] Jordan VC (1992) The strategic use of antiestrogens to control the development and growth of breast cancer. Cancer 70 (4 Suppl): :977–982.1638467

[3] HanahanD, WeinbergRA (2000) The hallmarks of cancer. Cell 100 (1): 57–70.1064793110.1016/s0092-8674(00)81683-9

[4] RochefortH, GlonduM, SahlaME, PlatetN, GarciaM (2003) How to target estrogen receptor-negative breast cancer? Endocr Relat Cancer 10 (2): 261–266.1279078710.1677/erc.0.0100261

[5] AndersC, CareyLA (2008) Understanding and treating triple-negative breast cancer. Oncology (Williston Park) 22 (11): 1233–1239.18980022PMC2868264

[6] GriffithsCL, OlinJL (2012) Triple negative breast cancer: a brief review of its characteristics and treatment options. J Pharm Pract 25 (3): 319–323.2255155910.1177/0897190012442062

[7] LiuD, HeJ, YuanZ, WangS, PengR, et al (2011) EGFR expression correlates with decreased disease-free survival in triple-negative breast cancer: a retrospective analysis based on a tissue microarray. Med Oncol 29 (2): 401–405.2126453110.1007/s12032-011-9827-x

[8] BadveS, DabbsDJ, SchnittSJ, BaehnerFL, DeckerT, et al (2011) Basal-like and triple-negative breast cancers: a critical review with an emphasis on the implications for pathologists and oncologists. Mod Pathol 24 (2): 157–167.2107646410.1038/modpathol.2010.200

[9] RobertsPJ, DerCJ (2007) Targeting the Raf-MEK-ERK mitogen-activated protein kinase cascade for the treatment of cancer. Oncogene 26 (22): 3291–3310.1749692310.1038/sj.onc.1210422

[10] HanH, DuB, PanX, LiuJ, ZhaoQ, et al (2010) CADPE inhibits PMA-stimulated gastric carcinoma cell invasion and matrix metalloproteinase-9 expression by FAK/MEK/ERK-mediated AP-1 activation. Mol Cancer Res 8 (11): 1477–1488.2104777010.1158/1541-7786.MCR-10-0114

[11] ShenQ, UrayIP, LiY, ZhangY, HillJ, et al (2008) Targeting the activator protein 1 transcription factor for the prevention of estrogen receptor-negative mammary tumors. Cancer Prev Res (Phila) 1 (1): 45–55.1913893510.1158/1940-6207.CAPR-08-0034PMC2577387

[12] BiswasDK, CruzAP, GansbergerE, PardeeAB (2000) Epidermal growth factor-induced nuclear factor kappa B activation: A major pathway of cell-cycle progression in estrogen-receptor negative breast cancer cells. Proc Natl Acad Sci U S A 97 (15): 8542–8547.1090001310.1073/pnas.97.15.8542PMC26984

RETRACTED

[13] KrolJ, FrancisRE, AlbergariaA, SuntersA, PolychronisA, et al (2007) The transcription factor FOXO3a is a crucial cellular target of gefitinib (Iressa) in breast cancer cells. Mol Cancer Ther 6 (12 Pt 1): 3169–3179.1808971110.1158/1535-7163.MCT-07-0507

[14] ZhangYG, DuQ, FangWG, JinML, TianXX (2008) Tyrphostin AG1478 suppresses proliferation and invasion of human breast cancer cells. Int J Oncol 33 (3): 595–602.18695891

[15] KimS, ChoiJH, KimJB, NamSJ, YangJH, et al (2008) Berberine suppresses TNF-alpha-induced MMP-9 and cell invasion through inhibition of AP-1 activity in MDA-MB-231 human breast cancer cells. Molecules 13 (12): 2975–2985.1905252210.3390/molecules13122975PMC6244848

[16] SaeedA, SharmaAP, DuraniN, JainR, DuraniS, et al (1990) Structure-activity relationship of antiestrogens. Studies on 2,3-diaryl-1-benzopyrans. J Med Chem 33 (12): 3210–3216.225890610.1021/jm00174a018

[17] United States Patent no. 5254,568; Inventors: RS Kapil, S. durani, JD Dhar, BS Setty; Title: Benzopyrans as anti-estrogenic agents.

[18] SharmaAP, SaeedA, DuraniS, KapilRS (1990) Structure-activity relationship of antiestrogens. Effect of the side chain and its position on the activity of 2,3-diaryl-2H-1-benzopyrans. J Med Chem 33: 3216–3222.225890710.1021/jm00174a019

[19] DharJD, SettyBS, DuraniS, KapilRS (1991) Biological profile of 2-[4-(2-N-piperidinoethoxy) phenyl]-3-phenyl(2H)benzo(b) pyran- a potent anti-implantation agent in rat. Contraception 44: 461–72.182455810.1016/0010-7824(91)90036-f

[20] SreenivasuluS, SinghMM, DwivediA, SettyBS, KambojVP (1992) CDRI-85/287, a novel antiestrogen and antiimplantation agent: biological profile and interaction with the estrogen receptors in immature rat uterus. Contraception 45: 81–92.159192510.1016/0010-7824(92)90144-i

[21] DwivediA, BansodeFW, SettyBS, DharJD (1999) Endometrial steroid receptors during decidualization in rhesus monkey (Macaca mulatta); their modulation by anti-oestrogen CDRI-85/287. Hum Reprod 14: 1090–1095.1022124610.1093/humrep/14.4.1090

[22] FatimaI, ChandraV, SaxenaR, ManoharM, SanghaniY, et al (2012) A 2,3-Diaryl-2H-1-benzopyran derivatives interfere with classical and non-classical estrogen receptor signaling pathways, inhibit Akt activation and induce apoptosis in human endometrial cancer cells. Mol Cell Endocrinol 348 (1): 198–210.2187836510.1016/j.mce.2011.08.018

[23] GuptaA, MandalSK, LeblancB, DescôteauxV, AsselinE, et al (2008) Synthesis and cytotoxic activity of benzopyran-based platinum(II) complexes. Bio Med Chem Lett 18: 3982–3987.10.1016/j.bmcl.2008.06.01318571403

RETRACTED

[24] BreschGJ, WolbergWH, GilchristKW, VoelkelJG, GouldMN (1983) A comparison of methods for the production of monodispersed cell suspensions from human primary breast carcinomas. Breast Cancer Res Treat 3 (1): 15–22.630743510.1007/BF01806230

[25] MorrisGM, HueyR, LindstromW, SannerMF, BelewRK, et al (2009) AutoDock4 and AutoDockTools4: Automated docking with selective receptor flexibility. J Comput Chem 30 (16): 2785–2791.1939978010.1002/jcc.21256PMC2760638

[26] SYBYL, version 7.3 (2006) Tripos Associates, St. Louis, MO, USA.

[27] WoodER, TruesdaleAT, McDonaldOB, YuanD, HassellA, et al (2004) A unique structure for epidermal growth factor receptor bound to GW572016 (Lapatinib): relationships among protein conformation, inhibitor off-rate, and receptor activity in tumor cells. Cancer Res 64 (18): 6652–6659.1537498010.1158/0008-5472.CAN-04-1168

[28] SeeligerD, de GrootBL (2010) Ligand docking and binding site analysis with PyMOL and Autodock/Vina. J Comput Aided Mol Des 24 (5): 417–422.2040151610.1007/s10822-010-9352-6PMC2881210

[29] MOE: The Molecular Operating Environment from Chemical Computing Group Inc, 1255 University St, Suite 1600, Montreal, Quebec, Canada H3B 3X3 (2012) Journal of Computer -Aided Molecular Design 26(6): 775-786 (last issue). Available: https://www.chemcomp.com/MOE-Structure_Based_Design.html.

[30] BlessonCS, AwasthiS, KharkwalG, DavereyA, DwivediA (2006) Modulation of estrogen receptor transactivation and estrogen-induced gene expression by ormeloxifene-a triphenylethylene derivative. Steroids 71 (11–12): 993–1000.1696579810.1016/j.steroids.2006.08.001

[31] XuYZ, ZhengRL, ZhouY, PengF, LinHJ, et al (2011) Small molecular anticancer agent SKLB703 induces apoptosis in human hepatocellular carcinoma cells via the mitochondrial apoptotic pathway *in vitro* and inhibits tumor growth *in vivo* . Cancer Lett 313 (1): 44–53.2194466110.1016/j.canlet.2011.08.025

[32] MelocheS, PouyssegurJ (2007) The ERK1/2 mitogen-activated protein kinase pathway as a master regulator of the G1- to S-phase transition. Oncogene 26 (22): 3227–3239.1749691810.1038/sj.onc.1210414

[33] DolcetX, LlobetD, PallaresJ, Matias-GuiuX (2005) NF-κB in development and progression of human cancer. Virchows Arch 446 (5): 475–482.1585629210.1007/s00428-005-1264-9

[34] HuMC, LeeDF, XiaW, GolfmanLS, Ou-YangF, et al (2004) IkappaB kinase promotes tumorigenesis through inhibition of forkhead FOXO3a. Cell 117 (2): 225–237.1508426010.1016/s0092-8674(04)00302-2

[35] EllerbroekSM, HalbleibJM, BenavidezM, WarmkaJK, WattenbergEV, et al (2001) Phosphatidylinositol 3-kinase activity in epidermal growth factor-stimulated matrix metalloproteinase-9 production and cell surface association. Cancer Res 61 (5): 1855–1861.11280738

RETRACTED

[36] LingH, ZhangY, NgKY, ChewEH (2011) Pachymic acid impairs breast cancer cell invasion by suppressing nuclear factor-kappaB-dependent matrix metalloproteinase-9 expression. Breast Cancer Res Treat 126 (3): 609–620.2052109910.1007/s10549-010-0929-5

[37] ChenPS, WangMY, WuSN, SuJL, HongCC, et al (2007) CTGF enhances the motility of breast cancer cells via an integrin-alphavbeta3-ERK1/2-dependent S100A4-upregulated pathway. J Cell Sci 120 (Pt 12): 2053–2065.1755097210.1242/jcs.03460

[38] ShimoT, KubotaS, YoshiokaN, IbaragiS, IsowaS, et al (2006) Pathogenic role of connective tissue growth factor (CTGF/CCN2) in osteolytic metastasis of breast cancer. J Bone Miner Res 21 (7): 1045–1059.1681352510.1359/jbmr.060416

